# Downregulation of X-linked inhibitor of apoptosis protein by ‘7-Benzylidenenaltrexone maleate’ sensitizes pancreatic cancer cells to TRAIL-induced apoptosis

**DOI:** 10.18632/oncotarget.17841

**Published:** 2017-05-12

**Authors:** So Young Kim, Sojung Park, SeonA Yoo, Jin Kyung Rho, Eun Sung Jun, Suhwan Chang, Kyung Kon Kim, Song Cheol Kim, Inki Kim

**Affiliations:** ^1^ ASAN Institute for Life Sciences, ASAN Medical Center, Seoul, 05505 South Korea; ^2^ Department of Convergence Medicine, University of Ulsan College of Medicine, Seoul, 05505, South Korea; ^3^ Department of Biomedical Sciences, University of Ulsan College of Medicine, Seoul, 05505, South Korea; ^4^ Division of HBP Surgery, Department of Surgery, University of Ulsan College of Medicine, Asan Medical Center, Seoul, 05505, South Korea

**Keywords:** BNTX, TRAIL, XIAP, PKCα, pancreatic cancer cells

## Abstract

Tumor necrosis factor-related apoptosis-inducing ligand (TRAIL) is a potential biological anticancer agent. However, a wide range of human primary cancers, including pancreatic cancer, display resistance to apoptosis induction by TRAIL. Therefore, this resistance needs to be overcome to allow TRAIL to be successfully used in cancer therapy. In this study, we performed a compound screen to isolate TRAIL sensitizers and found that one of the identified compounds, 7-benzylidenenaltrexone maleate (BNTX), sensitized pancreatic cancer cells to TRAIL-induced apoptotic cell death. The combination of BNTX with TRAIL promoted the release of cytochrome *c* from mitochondria into cytosol with caspase activation and a resulting increase in annexin V-stained cells. From a mechanistic perspective, we found that BNTX downregulated X-linked inhibitor of apoptosis protein (XIAP) expression when used in combination with TRAIL, and found that TRAIL-induced apoptosis was augmented by siRNA-mediated knockdown of XIAP. We further demonstrated that BNTX promoted the ubiquitin/proteasome-dependent degradation of XIAP protein via protein kinase C (PKC) alpha/AKT pathway inhibition. Moreover, combined treatment by BNTX with TRAIL suppressed growth of pancreatic tumor xenograft of animal model. Therefore, we suggest that inhibitor of apoptosis protein-mediated resistance of pancreatic cancer cells to anticancer therapeutics can be overcome by inhibiting the PKCα/AKT pathway.

## INTRODUCTION

Pancreatic cancer is a high-grade malignant tumor that is generally characterized by poor prognosis, with a 5-year survival rate of <5% [1]. Gemcitabine is the standard first-line therapeutic regimen as a single or combination treatment [2, 3]. However, the median overall survival of patients treated by gemcitabine is only 7.2 months [4]. Therefore, a new therapeutic approach is required to treat pancreatic cancer.

Tumor necrosis factor-related apoptosis-inducing ligand (TRAIL) is a proapoptotic cytokine that induces apoptosis only in cancer cells [5]. However, although human pancreatic cells have been shown to express TRAIL receptors, they are generally resistant to TRAIL-induced apoptosis [6]. The agonistic activation of TRAIL receptor by trimeric TRAIL results in upstream caspase-8 activation, which induces the activation of executioner caspases and the cleavage of Bid, initiating the apoptotic program [7].

The release of cytochrome *c* from mitochondria into cytosol triggers executioner caspase-3 activation via formation of the cytochrome *c*/caspase-9/Apaf-1 apoptosome complex, while Smac/DIABLO and HtrA2/Omi promote apoptosis by neutralizing inhibitors of apoptosis proteins (IAPs) [8]. The IAP protein family, which include XIAP, cIAP-1, cIAP-2, hILP-2, ML-IAP, NAIP, Apollon, and Survivin, are antiapoptotic regulators [9, 10], several of which have been shown to be upregulated in a wide range of cancers [11]. They are characterized by the protein domain ‘Baculovirus IAP repeat (BIR),’ which is responsible for inhibiting caspases [9, 12]. Of these IAPs, XIAP has been reported as the most potent inhibitory protein of apoptosis [11-15]. The role of XIAP in pancreatic cancer has been characterized by RNA interference technology [16, 17]. XIAP has three BIR domains, one ubiquitin-associated domain, and one really interesting new gene domain (RING), with E3 ubiquitin ligase activity implying that there is a complicated regulatory mechanism for this protein in cancer cells. Various studies have shown that IAPs are involved in the resistance of cancer cells to TRAIL [18]. However, the molecular mechanism controlling the resistance of pancreatic cancer cells to TRAIL-induced apoptosis via IAP has not yet been fully elucidated.

In this report, we performed a small scale high-throughput screening to identify the sensitizer of TRAIL-induced apoptosis in pancreatic cancer cells and investigated the underlying molecular mechanism of isolated sensitizer. We found that BNTX sensitized pancreatic cancer cells to TRAIL-induced apoptosis by downregulating XIAP via inhibition of the PKCα/AKT signaling pathway.

## RESULTS

### BNTX sensitizes pancreatic cancer cells to TRAIL-induced apoptosis

To characterize a novel survival pathway that regulates the resistance of pancreatic cancer cells to TRAIL, we performed high-throughput screening using a library of 1,280 biologically active compounds (LOPAC-1280^TM^). AsPC-1 cells were pre-treated with 5 μM library compounds for 1 h and then incubated with a sub-lethal dose of recombinant TRAIL (50 ng/ml) for an additional 24 h. Based on this screening, we defined a “sensitizer hit” as a compound that induced cell death in >50% of cells when combined with TRAIL, compared with a <15% cell death ratio in only 5 μM compound treated sample.

The primary screening showed that BNTX, a selective non-peptide delta 1(δ 1)-opioid receptor antagonist, sensitized AsPC-1 cells to TRAIL (Figure 1A). We confirmed that BNTX significantly enhanced TRAIL-induced cell death in a dose-dependent manner in combination with TRAIL (Figure 1B). Although we noted that higher concentrations of BNTX resulted in more profound cell death (40.3% at 20 μM), 5 μM BNTX slightly increased cell death to 10% compared with the control. To examine the specificity of molecular target involved in sensitization, we tested six additional opioid receptor antagonists for their TRAIL sensitization effect in AsPC-1 cells. Two of them (naloxone and naltrexone) are antagonists for various types of opioid receptors including μ, κ, and δ while the others (naltrindole, naltriben, ICI174864, and SDM25N) are δ type opioid receptor antagonists sharing similar target specificity with BNTX. From them only SDM25N induced statistically significant level of sensitization to TRAIL (Supplementary Figure 1A).

**Figure 1:** BNTX sensitizes human pancreatic cancer cells to TRAIL-induced apoptosis **(A)** Assay data for a screening analysis of AsPC-1 cells pre-incubated with various test compounds (5 μM) and were then exposed to TRAIL (50 ng/ml). Cell survival was measured as a percentage of the control sample. The arrow indicates BNTX (5 μM). **(B)** AsPC-1 cells were exposed to various concentrations of BNTX with or without TRAIL (25 ng/ml) for 24 h. Cell viability was measured by a luminescent CellTiter-Glo assay, and relative cell survival was determined by assaying ATP levels. **(C)** Relative survival of three pancreatic cancer cell lines (AsPC-1, PANC-1, and MIA PaCa-2) exposed to TRAIL (25 ng/ml) with or without BNTX (2.5 μM) for 24 h. Cell viability was measured by a luminescent CellTiter-Glo assay. **(D)** Apoptotic activity in AsPC-1 cells exposed to TRAIL (25 ng/ml) with or without BNTX (2.5 μM) for 24 h. Cells were analyzed by annexin V/PI double-stained flow cytometry. **(E)** The percentage of apoptotic cells. Values are the mean ± SD from two independent experiments performed in duplicate. Asterisks indicate significant differences compared with the control (*** P < 0.001). NS, not significant.

To further characterize the availability of BNTX as a sensitizer in pancreatic cancer cells, we examined its TRAIL-sensitizing effect in three pancreatic cancer cell lines (AsPC-1, PANC-1, and MIA PaCa-2). We found that BNTX reversed the resistance of all tested pancreatic cancer cells to TRAIL (Figure 1C).

For the qualitative analysis of sensitization, we used flow cytometry to detect apoptotic activity following combined treatment with BNTX and TRAIL. The combination of BNTX with TRAIL increased the annexin V positive cell population to 28.4 ± 2.8%, whereas there was no statistically significant increase in samples treated with either BNTX alone or TRAIL alone (Figure 1D and 1E).

### BNTX promotes TRAIL-induced apoptosis in a caspase-dependent manner

The molecular mechanism of BNTX-induced sensitization to TRAIL was examined by western blotting. We analyzed the expression of TRAIL receptor proteins (DR4 and DR5), activation of caspase, cleavage of poly (ADP-ribose) polymerase (PARP), and release of cytochrome *c* into the cytosol. As can be seen in Figure 2A, the individual treatment with BNTX or TRAIL did not induce any change in apoptotic cell signaling. Furthermore, the expression levels of TRAIL receptors were not altered by either a single or combination treatment. However, the combination of BNTX with TRAIL clearly led to the activation of caspase-3, -7, and -8; the cleavage of the caspase substrate PARP; and a profound release of cytochrome *c* from the mitochondria into the cytosol (Figure 2A). The involvement of caspases in this cell death was again examined by inhibitors. As shown in Figure 2B and 2C, caspase-3 inhibitor (z-DEVD-fmk) and caspase-8 inhibitor (z-IETD-fmk) were sufficient to suppress each enzyme activity (Figure 2B) and cleavage of caspase substrate (PARP) in combination treatment (Figure 2C). Taken together, these results indicate that BNTX sensitizes pancreatic cancer cells to TRAIL-induced apoptosis in a caspase-dependent manner.

**Figure 2:** BNTX induces TRAIL-induced apoptosis in AsPC-1 cells through caspase activation **(A)** Apoptosis signaling in AsPC-1 cells exposed to TRAIL (25 ng/ml) with or without BNTX (2.5 μM) for 24 h analyzed by western blot analysis using the indicated antibodies. The arrows indicate the cleaved forms of caspase-8 and PARP. M: mitochondrial fraction; C: cytosol fraction. **(B, C)** AsPC-1 cells were pre-treated with caspase inhibitors z-IETD-fmk (20 μM) or z-DEVD-fmk (20 μM) for 1h, and then exposed to BNTX (2.5 μM) with or without TRAIL (25 ng/ml) for 24 h. Cell lysates were performed to measure apoptosis by caspase activity (B) and western blot analysis for caspase-3,-8 and PARP (C). Values are the mean ± SD from two independent experiments performed in duplicate. Asterisks indicate significant differences compared with the control (*** P < 0.001).

### BNTX promotes the apoptotic program via XIAP downregulation, AKT pathway inactivation, and mitogen-activated protein kinase (MAPK) pathway activation

To understand the detail molecular mechanism of BNTX-induced sensitization, we analyzed changes in the expression and activity of apoptosis-related proteins in cells treated with BNTX, TRAIL, or a combination of the two. The combination of BNTX with TRAIL increased the expression of the proapoptotic proteins Bim and Bak and significantly decreased the expression of IAP proteins, including XIAP and Survivin (Figure 3A). However, no significant changes were observed in Bcl-2, Bcl-xL, Mcl-1, Bad, Bax, Puma, Noxa, and cIAP-1 proteins regardless of the treatment conditions. These findings suggest that the simultaneous regulation of proapoptotic Bcl-2 and antiapoptotic IAP proteins is a key mechanism in the sensitization of pancreatic cancer cells to TRAIL.

**Figure 3:** Effects of a combination of BNTX and TRAIL on the Bcl-2 protein family, IAP protein family, MAPKs, and AKT signaling molecules in AsPC-1 cells **(A, B)** AsPC-1 cells were exposed to TRAIL (25 ng/ml) with or without BNTX (2.5 μM) for 24 h, lysed, and analyzed by western blot analysis using the indicated antibodies. The results are representative of three independent experiments. The arrows indicate the three major isoforms of Bim, including BimEL, BimL, and BimS.

In the next step, we analyzed cell stress and survival signaling pathways, including MAPK and AKT. This included an examination of the phosphorylation of p38 MAPK and c-Jun at serine 73 and the activation of ERK and AKT. There was no significant change in cells treated with BNTX or TRAIL alone. However, western blot analysis showed that the combination of BNTX with TRAIL increased the phosphorylation of p38, c-Jun, and ERK but led to the dephosphorylation of AKT (Figure 3B).

In more detail, we examined whether p38, c-Jun, and ERK are involved in the apoptotic cell death induction by the combination of BNTX with TRAIL. In our test, all of p38 (SB202190), c-Jun (SP600125), and ERK (PD98059) inhibitors had no inhibitory effect on combined treatment-induced PARP cleavage (Supplementary Figure 2). Additionally, p38 and c-Jun inhibition did not block combined treatment-induced XIAP degradation. However, ERK inhibitor (PD98059) rather enhanced degradation of XIAP in combination treatment implying that ERK activation can serve a part of cancer cell survival signaling by protecting XIAP from degradation (Supplementary Figure 2C and 2D), while p38 and c-Jun associated signaling is not. These results, all together, indicate that combined treatment with BNTX and TRAIL triggers MAPK stress signaling but inactivates the AKT-mediated survival pathway.

### BNTX promotes ubiquitin/proteasome-dependent degradation of XIAP protein

To understand the detailed mechanism of BNTX-induced XIAP downregulation with sensitization to TRAIL, we further analyzed the effect of BNTX on XIAP expression. As shown in Figure 4A, the pre-incubation of cells with BNTX downregulated XIAP expression of protein in a dose-dependent manner, with the downregulation of XIAP being evident at BNTX concentrations of 5 and 10 μM. However, the downregulation of XIAP was further enhanced by combined treatment with BNTX and TRAIL (Figure 4A). XIAP downregulation was also accompanied by PARP cleavage (Figure 4A).

**Figure 4:** BNTX promotes the ubiquitin/proteasome-dependent degradation of XIAP in AsPC-1 cells **(A)** The expression of XIAP and cleavage of PARP in AsPC-1 cells exposed to various concentrations of BNTX with or without TRAIL (25 ng/ml) for 24 h was analyzed by western blot analysis. **(B)** The expression of XIAP, PARP, and caspase-3 cleavage in AsPC-1 cells transfected with scrambled control siRNA (siCont) or two different XIAP siRNAs (siXIAP#1 and siXIAP#2) for 48 h was analyzed by western blot analysis. **(C, D)** Transcriptional regulation of XIAP by a combination of BNTX (2.5 μM) and TRAIL (25 ng/ml) for 24 h was assessed using RT-PCR (**C**, upper panel), real-time qRT-PCR (**C**, lower panel), and the XIAP luciferase reporter assay **(D)**. Luciferase activity was measured by the luminescent dual-luciferase reporter assay and presented as the ratio of activity compared with the control. Values are the mean ± SD from three independent experiments performed in triplicate. Asterisks indicate significant differences compared with the control (** P < 0.01). NS, not significant. **(E)** The expression and phosphorylation of XIAP in AsPC-1 cells exposed to BNTX (10 μM) alone for the indicated time (upper panel) or pre-treated with MG132 (2.5 μM) for 1 h and then incubated with 10 μM BNTX for the indicated time (lower panel) were analyzed by western blot analysis. **(F)** Ubiquitination assays for AsPC-1 cells transfected with pcDNA3-Myc-XIAP and HA-Ub for 48 h, pre-treated with MG132 (2.5 μM) for 1 h, and then exposed to BNTX (10 μM) with or without TRAIL (25 ng/ml) for 3 h. Cell lysates were immunoprecipitated with Myc antibody and then detected using HA antibody (upper panel). Total cell lysates before immunoprecipitation (Input) were analyzed by western blot analysis using XIAP antibody (lower panel). Results are representative of three independent experiments.

The role of XIAP in apoptotic sensitization by BNTX was examined by knockdown and reconstitution assay. For the loss of function study, we knocked down XIAP with two different siRNAs and examined caspase activation by western blotting. Two siRNAs were successful in knocking down XIAP compared with the control siRNA, and both of these were also successful in sensitizing cells to TRAIL-induced cell death, as shown through the increased cleavage of caspase-3 and PARP (Figure 4B). For reconstitution of XIAP, we overexpressed wild type (HA-XIAP) or non-degradable XIAP mutant (HA-XIAP-S87D) in which serine 87 was replaced with aspartic acid, in AsPC-1 cells, followed by cell death evaluation and western blotting (Supplementary Figure 3A and 3B). Overexpression of XIAP successfully suppressed combination treatment-induced cell death with delayed caspase-3 activation (Supplementary Figure 3A). Moreover, reconstitution of XIAP by XIAP-S87D overexpression strongly inhibited combination treatment-induced cell death. The phospho-mimic pattern of XIAP-S87D, delayed degradation of XIAP and inhibited caspase activation were visualized by western blotting (Supplementary Figure 3B). Taken together, our results indicate that the downregulation of XIAP is one of the main mechanisms by which BNTX sensitizes cells to TRAIL.

To investigate how BNTX regulates XIAP protein expression, we first analyzed the effect of BNTX on XIAP mRNA transcriptional regulation using real-time RT-PCR and the dual-luciferase reporter assay. There were no statistically significant differences in XIAP mRNA levels and XIAP promoter luciferase activities between cells treated with BNTX alone or TRAIL alone and untreated cells. However, the combination of BNTX with TRAIL significantly increased XIAP mRNA levels by 4.14 ± 1.34 fold and increased XIAP promoter transcription levels by 10.9 ± 1.88 fold compared with untreated cells (Figure 4C and 4D). These findings raise the possibility that BNTX downregulates XIAP protein expression at the post-translational level. Therefore, because XIAP has been shown to possess E3 ubiquitin ligase activity and to be degraded by the proteasome system [19], we examined whether BNTX can trigger the ubiquitin/proteasome-dependent degradation of XIAP by assessing the phosphorylation status of XIAP at serine 87, which is a bypass signal that protects XIAP from degradation [20]. It was found that treatment with BNTX rapidly decreased XIAP phosphorylation at serine 87 in a time-dependent manner, with subsequent downregulated expression (Figure 4E, upper panels). Furthermore, although BNTX treatment decreased the phosphorylation of XIAP at the serine 87 residue, the total amount of XIAP remained at a similar level that of the control (Figure 4E, upper panels, lane 2). By contrast, the pre-treatment of cells with MG132, an inhibitor of the 26S proteasome, completely blocked BNTX-mediated XIAP downregulation (Figure 4E, lower panel), implying that BNTX triggered proteasome-mediated XIAP degradation.

The level of XIAP ubiquitination by BNTX was further examined using a XIAP-ubiquitination analysis. AsPC-1 cells were co-transfected with Myc-tagged XIAP and HA-tagged Ubiquitin, following which they were treated with MG132, BNTX, and TRAIL, as indicated in Figure 4F. Western blot analysis following immunoprecipitation revealed that there were no major changes in XIAP ubiquitination in the absence of MG132, regardless of treatment, whereas the total level of XIAP expression was downregulated by BNTX. By contrast, treatment with MG132 led to a profound increase in XIAP ubiquitination and a complete blocking of XIAP degradation in some samples (Figure 4F). Both TRAIL and BNTX individually increased ubiquitination of Myc-tagged XIAP protein, which was finally amplified by combination treatment (Figure 4F). These results indicate that a combination of BNTX with TRAIL amplified XIAP ubiquitination and induced XIAP degradation, which may be the main mechanism of BNTX-mediated TRAIL sensitization in pancreatic cancer cells.

### BNTX promotes TRAIL-induced apoptosis by XIAP downregulation via inhibition of the PKCα/AKT signaling pathway

It has previously been reported that AKT can interact with XIAP and phosphorylates it at serine 87, which serves as a protection mechanism against the ubiquitination and degradation of XIAP [19]. Therefore, to determine whether the BNTX-mediated downregulation of XIAP is dependent on the phosphatidylinositol 3-kinase (PI3K)/AKT signaling pathway, we analyzed the effect of PI3K inhibition on XIAP degradation in the presence or absence of BNTX and TRAIL.

Treatment with the PI3K inhibitor clearly decreased the AKT phosphorylation at serine 473 and downregulated XIAP expression (Figure 5A). However, the triple combination of BNTX with TRAIL in cells that had been pretreated with the PI3K inhibitor most significantly downregulated XIAP expression and increased the cleavage of caspase-3 and PARP (Figure 5A). These results suggest that the PI3K/AKT signaling pathway is involved in BNTX-mediated XIAP degradation and sensitization.

**Figure 5:** BNTX promotes XIAP downregulation by inhibiting the PKCα/AKT signaling pathway in TRAIL-treated AsPC-1 cells (A) The expression and phosphorylation of AKT, XIAP, PARP, and caspase-3 cleavage in AsPC-1 cells pre-treated with PI3K inhibitor (Wortmannin; 5 μM) for 0.5 h and then exposed to BNTX (2.5 μM) with or without TRAIL (25 ng/ml) for 24 h. Cell lysates were analyzed by western blot analysis using the indicated antibodies. (B) The expression and phosphorylation of PARP, XIAP, and AKT in two pancreatic cancer cell lines (PANC-1 and MIA PaCa-2) exposed to BNTX (2.5 μM) with or without TRAIL (25 ng/ml) for 24 h. Cell lysates were analyzed by western blot analysis using the indicated antibodies. The results are representative of three independent experiments. (C) The expression and phosphorylation of PKC, AKT, and XIAP in AsPC-1 cells exposed to TRAIL (25 ng/ml) with or without BNTX (2.5 μM) for 24 h, as determined by western blot analysis. (D) The expression and phosphorylation of AKT, XIAP, and PKC in AsPC-1 cells transfected with pHACE-HA-PKCα WT or pHACE-HA-PKCα DN (K368R) for 48 h, lysed, and analyzed by western blot analysis using the indicated antibodies. (E) The expression and phosphorylation of AKT and XIAP in AsPC-1 cells treated with the indicated concentrations of Go6976 for 24 h and analyzed by western blot analysis using the indicated antibodies. (F) The expression and phosphorylation of PKC and XIAP in AsPC-1 cells pre-treated with MG132 (2.5 μM) and/or Go6976 (10 μM) for 0.5 h and then exposed to BNTX (2.5 μM) with or without TRAIL (25 ng/ml) for 24 h were analyzed by western blot analysis. The results are representative of two independent experiments.

Next, we investigated whether XIAP downregulation in response to BNTX is a common event in pancreatic cancer cells by examining BNTX-mediated XIAP downregulation with AKT inactivation in PANC-1 and MIA PaCa-2 cells. In both lines, the combination of BNTX with TRAIL was successful in downregulating XIAP expression and increasing PARP cleavage, while AKT was inactivated, as revealed by the decreased phosphorylation at serine 473 (Figure 5B). Thus, BNTX-mediated XIAP downregulation appears to be a common event in pancreatic cancer cells.

In terms of the more upstream signaling of XIAP degradation, we reasoned that calcium-dependent kinase signaling may be involved. As already described, BNTX is aselective antagonist of the δ 1-opioid receptor, which triggers PKC-associated calcium signaling in the cell. Previous studies have shown that the phosphorylation of XIAP at serine 87 can be triggered by PKC in a similar way to AKT [20]; it has also been suggested that PKCα plays a role in the survival of pancreatic cancer cells [21, 22]. Therefore, we attempted to correlate PKCα and XIAP expression in TRAIL-induced apoptosis. As shown in Figure 5C, PKCα/β phosphorylation was not significantly affected by treatment with BNTX or TRAIL alone. However, combined treatment with BNTX and TRAIL significantly decreased the phosphorylation of PKCα/β, AKT, and XIAP. In this experiment, XIAP expression was downregulated as a result of decreased phosphorylation at serine 87.

Although we understood the involvement of AKT and PKCα in XIAP downregulation, the signaling between the two kinases remained unclear. Based on the findings of a previous study using myeloid progenitor cells [23], we hypothesized that the BNTX-induced suppression of PKCα activity causes AKT inactivation. To evaluate this possibility, we analyzed the effect of PKCα on AKT activation and XIAP phosphorylation. As shown in Figure 5D, the overexpression of wild-type PKCα significantly increased the phosphorylation of AKT and XIAP, whereas the overexpression of dominant-negative PKCα (K368R) decreased this. These data suggest that PKCα activates AKT, which induces XIAP phosphorylation to protect it from protein degradation. To investigate this possibility, we examined the effect of PKC inhibition on AKT activation and XIAP downregulation with XIAP phosphorylation. The PKCα/β inhibitor (Go6976) strongly inhibited the phosphorylation of AKT and XIAP in a dose-dependent manner (Figure 5E), indicating that PKC is involved in the protection of XIAP from protein degradation via the AKT pathway. Therefore, to confirm the detail role of PKC in XIAP degradation, we tested the effects of Go6976 on XIAP expression in combination with BNTX and TRAIL. We found that the combined treatment of Go6976 with BNTX/TRAIL decreased the phosphorylation of PKCα/β and completely enhanced the downregulation of XIAP. However, pretreatment with MG132 in the same experiment significantly restored XIAP from degradation (Figure 5F). These results suggest that PKCα-AKT signaling phosphorylates XIAP at serine 87 and that PKCα is one of the main regulators that controls XIAP protein degradation under a cell death-inducing environment in pancreatic cancer cells.

### Combined treatment with BNTX and TRAIL suppresses tumor growth and induces apoptosis *in vivo*

Finally, we examined the anticancer effects of combined treatment with BNTX and TRAIL *in vivo* using an AsPC-1 tumor xenograft model. Mice bearing implanted tumors were treated with BNTX, TRAIL, or a combination of the two. As shown in Figure 6A, combined treatment with BNTX and TRAIL suppressed the tumor volume compared with the control group or mice individually treated with each drug. Western blot analysis showed that the combination of BNTX with TRAIL reduced XIAP expression and increased caspase-3 and PARP cleavage in tumor tissue extracts after 20 days of treatment (Figure 6B). Immunohistochemical staining of the tumor tissues demonstrated a marked decrease in staining for Ki-67 in cells treated with a combination of BNTX and TRAIL, and a terminal deoxynucleotidyl transferase-mediated dUTP nick end labeling (TUNEL) assay also showed that the combination of BNTX and TRAIL statistically increased cell death compared with the control group or mice treated with TRAIL alone. All of these results suggest that combined treatment of BNTX with TRAIL suppresses tumor growth and induces apoptosis *in vivo*.

**Figure 6:** Combined treatment with BNTX and TRAIL induces tumor regression in a xenograft model **(A)** The mean tumor volumes in each treatment group. Asterisks indicate significant differences compared with the control (* *P <* 0.05). **(B)** The expression of XIAP, cleaved caspase-3, and PARP in protein extracts from tumor xenografts were analyzed by western blot analysis. **(C, D)** Representative images of tumor sections examined by immunohistochemical analysis (Ki-67 and TUNEL staining). The associated histograms show the number of immunopositive cells by the Ki-67 or TUNEL assay. Values are the mean ± SD (*n* = 5). Asterisks indicate significant differences compared with the control (** P < 0.01, *** P < 0.001).

## DISCUSSION

In this study, we identified BNTX as a new sensitizer for TRAIL in pancreatic cancer cells and elucidated the regulatory signaling pathway for molecular events involved in sensitization. Our data demonstrated that BNTX sensitized TRAIL-induced apoptosis in all tested pancreatic cancer cell lines, including AsPC-1, PANC-1, and MIA PaCa-2 (Figure 1C), by downregulating the expression of XIAP (Figure 3A). BNTX also synergistically worked with TRAIL to induce apoptosis in AsPC-1 cells via XIAP downregulation in a dose-dependent manner (Figure 4A), which was mediated by the inhibition of AKT (Figure 5A). A detailed mechanistic study showed that BNTX stimulates the ubiquitin/proteasome-dependent degradation of XIAP protein (Figure 4F) rather than suppressing the mRNA transcription of XIAP (Figure 4C and 4D). We found that XIAP was downregulated by BNTX via the ubiquitination/proteasome-dependent pathway, whereby XIAP degradation was completely blocked by proteasome inhibitors (Figure 4E) and the level of ubiquitylated XIAP was enhanced by combined treatment with BNTX and TRAIL (Figure 4F). These findings are consistent with those of previous reports showing that XIAP expression is regulated by the ubiquitin/proteasome system [19, 24]. We also characterized the role of the PKCα/AKT pathway in XIAP downregulation in AsPC-1 cells, which suggests that the inhibition of this pathway is an attractive target in pancreatic cancer therapy (Figure 5). In addition to PKCα/AKT pathway, we also suggest the possible mechanism where ERK can protect XIAP from BNTX-induced XIAP degradation signaling (Supplementary Figure 2C and 2D). Furthermore, we found that combined treatment with BNTX and TRAIL displayed antitumor activity in a xenograft model *in vivo* (Figure 6).

BNTX is a selective δ 1-opioid receptor antagonist [25], which reduces neurogenic ion transport mediated by opioid receptors in porcine ileal mucosa [26]. In our result, we have shown that two out of seven opioid receptor antagonists are effective to sensitize pancreatic cancer cells to TRAIL. These two (BNTX and SDM25N) compounds are similarly effective to antagonize δ-opioid receptors suggesting the possible role of δ-opioid receptors in cell death signaling (Supplementary Figure 1). δ-opioid receptors are membrane proteins with seven-transmembrane that couple to inhibitory G proteins such as Gαi and Gαo. BNTX has a potent antitussive effect by mediating the δ 1-opioid receptor but does not induce any physiological effect on the δ 2-opioid receptor [27, 28]. The activation of the opioid receptor has been shown to inhibit cAMP production via the suppression of the PKA and CREB signaling pathway. The cell survival pathway that involves δ-opioid receptor has been partially characterized in neuronal and cancer cells [29, 30], highlighting the relevance of the PI3K and MAPK pathways [31, 32]. By contrast, the inhibition of δ-opioid receptor has been shown to inhibit brain glioma cell proliferation and induce apoptosis via PKC inactivation [33]. However, the antitumor effect mediated by δ-opioid receptor and its mechanism of action in cancer cells have not yet been investigated.

XIAP expression has been shown to be associated with aggressive clinical behavior and disease progression in many cancers [34-37], and XIAP protein levels are correlated with the sensitivities of cells to cancer therapeutic agents such as nucleosides and cytarabine [38]. Consequently, several studies have inhibited XIAP to develop targeted cancer therapies [39, 40], and research has been conducted to determine delicate mechanisms for regulating XIAP proteins in cancer cells. To date, various cell signaling pathways for regulating XIAP proteins have been identified, including NF-κB- [41] and PI3K- [42] dependent mechanisms. The most important regulatory point for XIAP stability is the phosphorylation of serine 87, which is the bypass signal from proteasome-dependent degradation [19]. Originally, AKT has been reported to interact with and phosphorylate XIAP at serine 87, and this phosphorylation has been shown to inhibit cisplatin-induced apoptosis [19]. In addition, the serine 87 phosphorylation of XIAP by PKC has been identified during DNA damage-induced apoptosis signaling [20]. These findings raised the possibility that the PKC-AKT axis is involved in the regulation of XIAP protein stability. However, the role of the PKCα-AKT pathway in pancreatic cancers remains unclear at the molecular level. Thus, to our knowledge, our study is the first to provide evidence on XIAP regulation by the PKCα-AKT axis in pancreatic cancers.

In terms of the relationship between δ-opioid receptors and PKC, it has previously been reported that the inhibition of δ-opioid receptors induces brain glioma cell apoptosis by inactivating PKC [33]. Thus, we hypothesized that antagonization of the δ 1-opioid receptor by BNTX downregulates XIAP expression via a coordinated regulatory mechanism between PKC and AKT signaling. Our data supported this, showing that BNTX treatment inhibited the phosphorylation of PKCα with inactivation of AKT (Figure 5C) and that this inactivation resulted in the dephosphorylation of XIAP at serine 87 with proteasome-dependent degradation (Figure 5F). Furthermore, this result was supported by our finding that wild-type PKCα induced serine 87 phosphorylation, while dominant-negative PKCα reversed this effect (Figure 5D).

To our knowledge, our study is the first to provide evidence that the combination of BNTX with TRAIL synergistically induces apoptosis by downregulating XIAP in pancreatic cancer cells and that this effect is mediated by the inhibition of the PKCα and AKT pathways. BNTX promoted the ubiquitin/proteasome-dependent degradation of XIAP protein in AsPC-1 cells. These findings indicate that the inhibition of δ-opioid receptors induces cancer cell apoptosis via XIAP regulation and provide a rationale for further developing the use of TRAIL to inhibit δ-opioid receptors and overcome apoptosis resistance in various human cancer cells.

## MATERIALS AND METHODS

### Cell culture and reagents

AsPC-1, PANC-1, and MIA PaCa-2 human pancreatic cancer cells were purchased from American Type Cell Culture (Manassas, VA). All cells except AsPC-1 were maintained in Dulbecco’s modified Eagle’s medium supplemented with 10% fetal bovine serum,_L_-glutamine, and 100 U/ml of antibiotic penicillin/streptomycin (all purchased from Life Technologies (Carlsbad, CA). AsPC-1 cells were maintained in RPMI-1640 with the same supplements. All cells were cultured at 37°C in a humidified atmosphere with 5% CO_2_. BNTX maleate salt hydrate and wortmannin were purchased from Sigma Aldrich (St. Louis, MO); Go6976 and MG132 were purchased from Calbiochem (San Diego, CA). Protein G agarose beads and recombinant human TRAIL were purchased from Life Technologies (Carlsbad, CA).

### Compound screening

The compound screening method used to identify the sensitizers of TRAIL in AsPC-1 cells has been previously described [43]. Cells were recovered from the culture and re-plated in cell culture grade lumitrac 96-well plates at a density of 5 × 10^3^ cells/well in 50 μl tissue culture medium. Using a liquid handler (Janus: Perkin-Elmer model), 25 μl of culture medium harboring library compound was transferred to the wells achieving final 5 μM concentration. After 1 h of pre-incubation, 25 μl of TRAIL-containing medium was injected to each well to yield final 50 ng/ml TRAIL concentration. After 24 h, the luminescence produced by ATP reaction of each well was measured by CellTiter-Glo assay solution (Promega) and a Victor Multi-label counter (Perkin-Elmer). Raw values were transferred to Prism software to evaluate relative cell survival. The library of biologically active compounds (LOPAC 1280^TM^; Sigma Aldrich, St. Louis, MO) was used in this study.

### Western blot analysis

Cell extracts were prepared by adding a lysis buffer [20 mM Tris-HCl (pH 7.5), 150 mM NaCl, 1 mM EGTA, 1mM EDTA-2Na), 1% Triton-X 100, 2.5 mM sodium pyrophosphate, 1 mM β-glycerophosphate, 1 mM Na_3_VO_4_, and 1 µg/ml leupeptin] containing complete protease and phosphatase inhibitor cocktails (Roche, Basel, Switzerland). After measuring protein concentrations using the bicinchoninic acid protein assay (Pierce, Rockford, IL), extracts were diluted in a 5 × Laemmli sample buffer, following which a 20 μg cell extract was resolved by sodium dodecyl sulfate-polyacrylamide gel electrophoresis (SDS-PAGE) and transferred to polyvinylidene difluoride (PVDF) membranes (Millipore, Billerica, MA). These were then incubated with the following primary antibodies (1:1000 dilutions): anti-p-AKT (#4060), anti-AKT (#4691), anti-Bad (#9292), anti-Bak (#6947), anti-Bax (#2772), anti-Bcl-2 (#2872), anti-Bcl-xL (#2764), anti-Bim (#2933), anti-cleaved caspase-3 (#9665), anti-caspase-7 (#9494), anti-caspase-8 (#9746), anti-cIAP-1 (#7065), anti-DR5 (#8074), anti-p-c-Jun (#9164), anti-p-p38 (#9216), anti-p38 (#9212), anti-p-ERK (#4370), anti-ERK (#4695), anti-HA (#3724), anti-Mcl-1 (#5453), anti-Myc (#2276), anti-p-PKCα/β II (#9375), anti-PARP (#9532), anti-Survivin (#2808), anti-Ubiquitin (#3936), and anti-XIAP (#2045), which were purchased from Cell Signaling Technology (Danvers, MA); anti-Puma (AB-33906), which was purchased from Abcam (Cambridge, MA); anti-DR4 (sc-7863), anti-PKCα (sc-8393), anti-c-Jun (sc-1694), and anti-Noxa (sc-30209), which were purchased from Santa Cruz Biotechnology (Santa Cruz, CA); and anti-p-XIAP (SAB4301454) and anti-α-Tubulin (T9026), which were purchased from Sigma Aldrich (St. Louis, MO).

Cytochrome *c* release from the mitochondria was analyzed with the Cytochrome c Releasing Apoptosis Assay Kit (GTX-85531; GeneTex, Irvine, CA). Primary antibodies were recognized using the horseradish peroxidase-conjugated goat anti-rabbit or goat anti-mouse secondary antibody (Cell Signaling, Danvers, MA), and protein bands were visualized by an enhanced chemiluminescent substrate solution (SuperSignal West Pico; Pierce, Rockford, IL).

### Cell viability assay and flow cytometry

Cells were seeded at 2∼3 × 10^3^ cells/well in 96-well plates and were pre-treated with BNTX at indicated concentrations for 0.5 h followed by TRAIL (25 ng/ml) for an additional 24 h. Cell viability assays were performed using a cellular ATP-based luminescence assay kit (CellTiter-Glo; Promega, Madison, WI). The raw value was analyzed using GraphPad Prism (La Jolla, CA) to evaluate the relative cell survival rate. The induction of apoptosis was determined using an Alexa Fluor® 488 Annexin V apoptosis kit (Invitrogen, Carlsbad, CA), according to the manufacturer’s instructions. Briefly, AsPC-1 cells were seeded in 60 mm dishes at 70 % confluence and harvested following treatment with BNTX (2.5 μM) and TRAIL (25 ng/ml) for 24 h. They were then stained with an Annexin V buffer containing an Annexin V and a propidium iodide solution (50 μg/ml). The percentage of apoptotic cell population was detected by flow cytometry analysis using a FACS Calibur analytical instrument (BD Biosciences, San Jose, CA).

### Caspase activity assay

The activity of caspase-3 and -8 were measured using a colorimetric assay system (R&D system, MA, USA) according to the manufacturer’s instructions. After 1 h of pre-incubation with caspase inhibitor, cells were exposed to BNTX (2.5 μM) with or without TRAIL (25 ng/ml) for 24 h. Cells were harvested using lysis buffer, after which cell lysates were incubated with caspase-3 (DEVD-pNA) or caspase-8 (IETD-pNA) substrate for 2 h at 37°C. The absorbance at 405 nm was measured with a spectrometer.

### Dual-luciferase activity assay

AsPC-1 cells were seeded at a density of 4 × 10^5^ cells in 6-well plates and were co-transfected with expression plasmids containing luciferase reporter (pGL2-XIAP-luc and pRL-TK-luc) using Lipofectamine® 2000 reagent (Invitrogen, Carlsbad, CA) for 48 h. Cells were then pre-incubated with BNTX (2.5 μM) for 0.5 h, following which they were exposed to TRAIL (25 ng/ml) for an additional 24 h. Following treatment, cells were lysed with the lysis buffer, and the transcription levels of XIAP were analyzed using a Dual-Luciferase Reporter Assay kit from Promega (Madison, WI). At least four independent experiments were performed in triplicate, and firefly luciferase activity was normalized to Renilla activity. pGL2-XIAP-luc promoter plasmids were kind gift from Dr. Yong-Sung Juhnn (Seoul National University College of Medicine, Korea).

### Expression constructs and siRNA transient transfection

AsPC-1 cells were transfected with pHACE-HA-PKCα WT or pHACE-HA-PKCα DN (K368R) plasmids (Addgene, Cambridge, MA) for 48 h using Lipofectamine® 2000 (Invitrogen, Carlsbad, CA), according to the manufacturer’s protocol. Cells were then lysed and analyzed by western blot analysis. XIAP siRNAs (#1: 5′-GAAGGAGAUACCGUGCGGUGCUUUA-3′; #2: 5′-CCAGAAUGGUCAGUACAAAGUUGAA-3′) and a control siRNA (5′-ACGUGACACGUUCGGAGAAUU-3′) were purchased from Dharmacon (Lafayette, CO). AsPC-1 cells were seeded at a density of 4 × 10^5^ cells in 6-well plates and were transiently transfected by 30 pmol siRNA with 5 μl RNAiMAX^TM^ (Life Technologies, Carlsbad, CA). After 48 h incubation, cells were treated with TRAIL (25 ng/ml) for an additional 24 h, and the gene knockdown efficiency of each sample was confirmed by western blotting. The XIAP reconstitution experiment was performed by same procedure with PKC. The expression plasmids of XIAP were kindly gifted by Dr. Duckett Colin Stephen, Baylor College of Medicine (HA-XIAP) and Dr. Donghoon Jin, University of Ulsan College of Medicine (HA-XIAP-S87D).

### Quantitative RT-PCR (qPCR)

Total RNA was extracted using the TRI Reagent® (Molecular Research Center, Cincinnati, OH), and cDNA was obtained using a RevertAid First Strand cDNA Synthesis Kit (Life Technologies, Carlsbad, CA). XIAP mRNA expression was analyzed using a LightCycler® 480 instrument (Roche Diagostics Ltd, Burgess Hill, UK) with SYBR® Green Master Mix. The following primer sequences were used for qPCR: XIAP, (sense) 5′-CCGTGCGGTGCTTTAGTTGT-3′ and (antisense) 5′-TTCCTCGGGTATATGGTGTCTGAT-3′ and GAPDH, (sense) 5′-GAGTCAACGGATTTGGTCGT-3′ and (antisense) 5′-TTGATTTTGGAGGGATCTCG-3′. The real-time qRT-PCR protocol was as follows: 95°C for 5 min, followed by 40 cycles at 95°C for 10 s, 58°C for 20 s, and 72°C for 10 s. The relative concentrations of PCR products were analyzed using the LightCycler® 480 System software (Roche Diagostics Ltd, Burgess Hill, UK). At least three independent experiments were performed in triplicate, and all samples were normalized to GAPDH.

### Immunoprecipitation and ubiquitination assay

AsPC-1 cells (5 × 10^6^) were transfected with plasmids encoding pcDNA3-Myc-XIAP and HA-Ub using Lipofectamine® 2000 for 48 h. Cells were pre-incubated with 2.5 μM MG132 for 1 h and then treated with BNTX (10 μM) and TRAIL (25 ng/ml) for 3 h. They were then lysed with an IP buffer [20 mM Tris-HCl (pH 7.5), 150 mM NaCl, 1 mM EGTA, 1 mM EDTA, 1% NP-40, 2.5 mM sodium pyrophosphate, 1 mM β-glycerophosphate, 1 mM Na_3_VO_4_, and 1 µg/ml leupeptin] containing complete protease and phosphatase inhibitor cocktails (Roche, Basel, Switzerland) for 0.5 h. After centrifugation, cell lysates were incubated with anti-Myc antibody (1 μg) overnight at 4°C on a rotator and then incubated with Protein G agarose beads (100 μl) for 2 h. Following a second centrifugation, the cell pellet was washed three times with the lysis buffer and boiled with a 2 × Laemmli sample buffer for 5 min. The ubiquitination of Myc-XIAP protein was detected by western blotting using anti-HA antibody.

### *In vivo* xenograft model

All experimental procedures were conducted following a protocol approved by the Institutional Animal Care and Use Committee of Asan Institute for Life Sciences (Permit Number: 2015-12-087, Seoul, Korea). All efforts to minimize suffering were made in this experiment. To establish a xenograft model, male nude mice (6∼8 weeks of age) were purchased from Charles River Laboratories (Wilmington, MA). Tumors were grown by implanting cells (1 × 10^6^ cells/0.1 ml) in 50% matrigel (BD Biosciences, San Jose, CA) and were subcutaneously injected into the right flank of each animal. When the tumor volume reached approximately 100 mm^3^, the mice were divided into four treatment groups (*n* = 5 per group): untreated, TRAIL (10 mg/kg), BNTX (0.5 mg/kg), and combination of BNTX (0.5 mg/kg) and TRAIL (10 mg/kg). Both TRAIL and BNTX were dissolved in a HEPES buffer. All drugs were administered by an intraperitoneal injection twice a week. To assess tumor size, the length (*L*) and width (*W*) of each tumor was measured using calipers, and the tumor volume (TV) was calculated as TV = (*L* × *W*^2^)/2. Lysates were prepared from tumor tissues, and protein levels were detected by western blotting using anti-XIAP, anti-cleaved caspase-3 and anti-PARP antibodies.

### Immunohistochemical staining

Each tumor was harvested at the indicated times post drug administration. Resected tumors were fixed in 10% formaldehyde and embedded in paraffin. Immunohistochemical staining was performed using a specific primary antibody [anti-Ki-67 (TEC-3) antibody; DakoCytomation, Los Angeles, CA], an EnVision Plus staining kit (DakoCytomation), and an APO-Direct TUNEL assay kit (Millipore, Temecula, CA), according to the supplier’s instructions. The quantitative analysis of section staining was performed by counting the number of immune-positive cells in five arbitrarily selected fields.

### Statistical analysis

All data were obtained from at least two or three independent experiments and are presented as the mean ± SD. Treatments were compared using two-way analysis of variance in GraphPad Prism 5.0. *** *P* < 0.001, ** *P* < 0.01, and * *P* < 0.05 were considered statistically significant.

## SUPPLEMENTARY MATERIALS FIGURES



## Abbreviations

BIR: Baculovirus IAP repeat
BNTX: 7-benzyl-idenenaltrexone maleate
IAP: inhibitor of apoptosis protein
MAPK: mitogen-activated protein kinase
PI3K: phosphatidylinositol 3-kinase
PARP: poly (ADP-ribose) polymerase
PKC: protein kinase C
TRAIL: tumor necrosis factor-related apoptosis-inducing ligand
TUNEL: terminal deoxynucleotidyl transferase-mediated dUTP nick end labeling
XIAP: X-linked inhibitor of apoptosis protein
